RETRACTED

# Immunomodulatory Effect of *Lycium barbarum* Polysaccharides against Liver Fibrosis Based on the Intelligent Medical Internet of Things

**DOI:** 10.1155/2022/6280265

**Published:** 2022-01-25

**Authors:** Yanzhen Han, Yan Zhou, Tieying Shan, Wei Li, Haiping Liu

**Affiliations:** ^1^General Surgery, Affiliated Hospital of Hebei University of Engineering, Handan 056002, Hebei, China; ^2^Medical College, Hebei University of Engineering, Handan 056002, Hebei, China; ^3^International Exchange College, Hebei University of Engineering, Handan 056002, Hebei, China; ^4^General Surgery, Handan Central Hospital, Handan 056002, Hebei, China

## Abstract

*Lycium barbarum* polysaccharide (LBP) is the main active component of *Lycium barbarum* and has many beneficial effects, including neuroprotection, antiaging, and antioxidation. This study mainly explores the immunomodulatory effect of *Lycium barbarum* polysaccharides against liver fibrosis based on the intelligent medical Internet of Things. This measure emphasizes that the current effective methods and methods for the treatment of liver cancer are mainly combined treatments of Western medicine and Chinese medicine. These treatments have a certain effect in preventing liver cancer, reducing recurrence, and reducing side effects. Among them, chemotherapy has unique advantages in improving the quality of life and prolonging survival. With the development of medical science and technology, the clinical efficacy and efficacy of traditional Chinese medicine in the treatment of liver cancer are constantly improving. The mechanism is also studied from many aspects. The treatment time of LBPs on fibrotic hepatocytes was set to 24 h. Take liver fiber cells in logarithmic growth phase and incubate them at 37°C for 24 h. The whole process uses a temperature sensor for intelligent temperature control. In the experiment, groups of LBPs with different concentrations and different molecular weight ranges were set up and each group had 6 multiple holes. The original medium was aspirated and replaced with a medium containing different concentrations of LBPs (12.5, 25, 50, 100, and 200 *μ*g/mL) and cultured for 24 h. Based on the previous research, this study used in vitro cell experiments, microscopic observation, and MTT method to verify whether *Lycium barbarum* polysaccharides inhibit the proliferation of human liver cancer cells in vitro and whether they cooperate with the chemotherapy drug fluorouracil to play a tumor-killing effect. Animal experiments, using ELISA, HE staining, and other methods, explore the molecular and immunological mechanisms of LBP's antiliver cancer effect from the perspective of Th/Th2 differentiation balance and DC function, in order to provide experimental evidence for Chinese medicine polysaccharides in cancer immunotherapy and application. At different LBP concentrations (0 *μ*mol/L, 5 *μ*mol/L, 10 *μ*mol/L, and 15 *μ*mol/L), the inhibition rates were 0.80%, 20.06%, 35.44%, and 55.39%, respectively. This study provides a new method for large-scale expansion of hepatocytes in vitro, laying a stronger foundation for biological treatment of liver fibrosis.

RETRACTED

## 1. Introduction

Tumor is a kind of common and frequently occurring disease that seriously harms human physical and mental health, among which malignant tumor is particularly serious. Worldwide, the incidence and mortality of cancer are increasing year by year. More than 7 million people die from malignant tumors every year. In some countries in Europe and the United States, the death rate of cancer is second only to cardiovascular diseases. Due to the histological and anatomical characteristics of the liver itself, primary liver cancer is an extremely aggressive malignant tumor. Most patients are already in the middle and late stage when they are treated, and most patients are accompanied by cirrhosis, hepatitis, and the resulting liver function damage. As a result, the average survival time of patients who cannot be treated is only 3-4 months, and the prognosis is extremely poor. Malignant tumors have become the most severe and urgent public health problem in the world due to their consistently high morbidity and mortality characteristics. Cancer deaths account for a quarter of all deaths. It has had a great destructive effect on human life and health. Factors that increase the risk of PHC (primary liver cancer) include long-term, heavy drinking and chronic infection with hepatitis B or C virus [1].

Although the level of diagnosis and treatment of liver cancer is constantly improving, the incidence and mortality of liver cancer are still high. The theoretical therapeutic potential of gene immunotherapy, which is considered as the most promising method in recent years, has not been fully realized. Liver transplantation is considered to be the most satisfied with the treatment, but difficult graft source and postoperative recurrence of problems, so liver transplantation is limited to the treatment of small tumors: early surgical resection does not change because of the large mass associated with recurrence of liver lesions, internal, anesthesia and surgery, liver blood flow blocking, and ischemia-reperfusion injury resulting in further suppressed immune function may cause cancer and further deterioration of the disease development. Liver transplantation is currently the most effective method, but the source of the liver, the cost of the operation, postoperative rejection, and recurrence make the transplantation operation not popular. Primary liver cancer (PHC) ranks sixth in the world among all cancers. Due to the increasing number of patients with liver fibrosis and alcoholic fatty liver (AFL) being its early reversible disease stage, therefore, the in-depth study of AFL is particularly important. Because primary liver cancer surgery resection rate is only 10% or so and postoperative recurrence rate is high, a variety of nonsurgical therapy remains: the main treatment of primary liver cancer, such as system and hepatic arterial infusion chemotherapy and embolization chemotherapy and radiotherapy (including radio frequency ablation or alcohol), have more severe immune and hematopoietic function of inhibiting and other side effects. Liver fibrosis is a compensatory response secondary to liver inflammation or tissue repair after injury. It is the common pathological basis of all chronic liver diseases and the main intermediate link in the development of liver cirrhosis. Its essence is the ECM when the tissue repair reaction occurs. The pathological process caused by the imbalance of synthesis, degradation and deposition, and liver fibrosis can eventually develop into liver cirrhosis and even liver cancer. Liver fibrosis and liver cirrhosis seriously affect human health. How to block the process of liver fibrosis is currently the focus of attention. This study uses smart medicine and *Lycium barbarum* polysaccharides to treat liver fibrosis, which has important clinical guiding significance.

RETRACTED

At present, the treatment measures for liver cancer emphasize the implementation of comprehensive treatment, that is, through the combination of western medicine, traditional Chinese medicine, and other effective means and methods (such as cancer gene therapy and biological therapy). Traditional Chinese medicine has unique advantages in preventing the occurrence of liver cancer, reducing recurrence, alleviating the toxic and side effects of radiotherapy and chemotherapy, improving the quality of life, and prolonging survival. With the development of medical science and technology, the clinical efficacy of traditional Chinese medicine in treating liver cancer has been continuously improved, and the research on the mechanism of drug action has been carried out from many aspects. Wolfberry has been used as a traditional medicinal herb and food supplement in China for more than 2,000 years. *Lycium barbarum* is rich *in Lycium barbarum* polysaccharides (LBP), betaine, phenols, cerebrosides, 2-O-*β*-d-glucopyranosyl-l-ascorbic acid (AA-2*β*G), flavonoids, and vitamins. LBPs are the main active ingredients of wolfberry. Gao discussed the pharmacological activities of LBP and other main ingredients. They mediate significant antiaging effects through antioxidant, immunomodulatory, antiapoptotic activity, and reduction of DNA damage. Therefore, basic scientific evidence for the antiaging effects of LBPs is already available. However, more research is needed to understand the mechanism by which LBP mediates antiaging properties. The new findings of his research may pave the way for the clinical application of Chinese medicine wolfberry in modern evidence-based medicine [2]. Zhang's research aimed to determine whether *Lycium barbarum* polysaccharides (LBPs) can protect mice from cadmium- (Cd-) induced testicular toxicity. The four groups were given oral cadmium chloride (5.0 mg/kg body weight) for 35 days and combined treatment with LBPs (0, 10, 33.3, or 100 mg/kg), from the week before exposure to Cd until the end of the experiment. The other two groups were given oral administration only with vehicle or LBP (100 mg/kg). LBP pretreatment improved the decrease in body weight, sperm motility, and serum testosterone levels caused by Cd. In addition, cadmium-induced abnormal sperm increase decreased, and LBPs effectively attenuated Cd-induced degeneration of seminiferous tubules. Therefore, LBPs can reduce Cd-induced testicular damage by improving antioxidant enzyme activity and reducing oxidative stress, so it may be a potential adjuvant therapy for Cd-induced testicular toxicity [3]. Masci A. believes that in the past few decades, the sugar compound from the fruit of wolfberry (*Lycium barbarum*) has received great attention due to its potential health promotion effect. His review included investigations on the extraction and purification methods of these biologically active molecules (LBPs), as well as studies on the structural characteristics of carbohydrate components. In addition, an overview of in vitro, in vivo, and clinical studies on the hypoglycemic and hypolipidemic effects of the isolated LBP components is reported. In his research, these purified components of wolfberry fruit may be potentially useful as an adjuvant treatment of diabetes and related diseases [4]. Li et al. believe that due to the modern sedentary and food-rich lifestyle, nonalcoholic fatty liver disease (NAFLD) is one of the main causes of chronic liver disease around the world. Autophagy is the protective self-digestion of intracellular organelles, including lipid droplets (fat phagocytosis), to maintain homeostasis in response to stress. In addition to lipolysis, fat phagocytosis is another way of lipid degradation. Impaired autophagy can also help treat NAFLD. Treatment with traditional Chinese herbal extracts may improve NAFLD. Their review will deeply explore the characteristics of autophagy in NAFLD and the traditions of resveratrol, wolfberry polysaccharides, dioscin, bergamot polyphenol components, capsaicin, and garlic derived S-allyl mercaptocysteine. The relevant actions/mechanisms of Chinese herbal extracts in inducing autophagy may inhibit the progression of NAFLD. In this research, the use of traditional Chinese herbal extracts to regulate autophagy/lipid autophagy may be a new method for the treatment of NAFLD, and its molecular mechanism should be further elucidated in the near future [5]. Yu et al. and Abdel-Basset et al. believes that the mechanism by which LBP prevents cerebral ischemia/reperfusion injury is still unclear. In addition, LBP was significantly reduced, and OGD/R induced apoptosis and autophagic cell death. LBP leads to the downregulation of cleaved caspase 3/caspase 3, LC3II/LC3I, and beclin 1, as well as the upregulation of Bcl-2/Bax and p62. In his research, only further analysis of the experiment was carried out, and the necessary research data was lacking [6, 7]. The body's antitumor immune relies mainly on T cell-mediated immune cells, T lymphocyte counts, the group of imbalance, and T lymphocyte activation barriers; increased apoptosis which is the main performance of the a tumor-burdened organism cellular immune function is low, and T lymphocytes in tumor local immune microenvironment and inhibition of function can directly reflect the body's antitumor cellular immune function.

RETRACTED

T cell activation requires at least two signals. The first signal is the interaction between the specific antigen recognition receptor (TCR) on the surface of T cells and the antigen binding MHC complex on the antigen-presenting cells (tumor cells or macrophages, dendritic cells, etc.). The second signal is coordinated stimulus on the antigen-presenting cells and T cells in the corresponding receptors. There are a lot of synergy to stimulate molecules involved in T cell activation, such as cell adhesion molecules (ICAMs), vascular cell adhesion molecule (VCAMs), lymphocyte function associated antigen 3 (LFA-3), and heat shock protein, and no second signal of synergy. In this study, a mouse liver fibrosis model was constructed to further investigate the effects of different molecular weight LBP components on the growth of mouse fibrotic cells and the immune system from in vivo experiments. Liver fibrosis is continuously formed in the proliferation of cancer cells or the metastasis of signal transmission pathways in various ways under the action of multiple factors. The tumor microenvironment is complicated, and single treatment or drugs cannot effectively control the onset of liver cancer. Therefore, investigating methods and drug combination therapy is a new strategy for the treatment of liver cancer. This study focused on the early stage of steatosis of alcoholic liver disease, clarified the effect of ethanol on ALT, AST, and lipid peroxidation, further verified its etiology, and investigated the prevention and treatment of AFL and its molecular mechanism by LBP Effectiveness.

RETRACTED

## 2. Research Methods

### 2.1. Cell Experiment Materials

#### 2.1.1. Cell Lines and Culture Methods

The liver fiber cell line of human liver cancer was gifted by the medical school and preserved by the Biochemical Pathology Research Group of the University of Traditional Chinese Medicine. After the cells were resuscitated, they were subcultured in a medium incubator with (RPMI 1640 + 10% calf serum + 1% penicillin) for subsequent experiments.

#### 2.1.2. Drugs and Reagents

Cell culture flasks, Pasteur pipettes, 96-well plates, 6-well plate culture plates, cryopreservation tubes, and so on are products of Nest company. Microporous membranes are purchased from Corning; syringes, medical cotton, and so on are purchased from Minkang Medical Equipment Co., Ltd. PBS buffer and pancreatin are prepared by our laboratory. PBS preparation method is as follows: weigh 8 g NaCll, 0.2 g KCll, 0.2 g KH_2_P0_4_, and 7.84 g Na_2_HP0_4_ (12H_2_0) into pure water and stir to dissolve the volume to 1 L and adjust the pH to 7.2–7.4 and high pressure of 0.22 *μ*m after sterilization.

Pore size microporous filter filtration is as follows. In pancreatin preparation method, add 0.25 g pancreatin and 0.02 g EDTA to 0 and IL of PBS to fully dissolve and then slowly stir overnight at 4°C and pH value (7.2–7.4), and use 0.22 *μ*m microporous filter and cryopreserve.

#### 2.1.3. Instruments and Equipment

Inverted phase contrast fluorescence microscope (Siemens, Germany), cell incubator (Invitrogen, US), cell cryopreservation tube (ABC, US), electric heating constant temperature water bath (Invitrogen, US), medical ultraclean workbench (Sigma, US), high-speed low-temperature desktop centrifuge (Invitrogen, USA) fluorescence quantitative PCR instrument, and horizontal electrophoresis equipment (BIO-RAD) were used.

### 2.2. Preparation of Experimental Drugs

Use an analytical balance to weigh 40 mg of *Lycium barbarum* polysaccharide powder, dissolve it in 8 mL of saline, mix well, and put it in a 10 mL EP tube and store it at 4°C. For cyclophosphamide injection, first use a syringe to inject 10 mL of normal saline into the bottle, shake it completely before the solution becomes transparent, and then prepare 0.29/mL of mother liquor. It can be used immediately, stored at 4°C for a short period of time, and then frozen at −20°C for a long time. The whole process uses a temperature sensor for intelligent temperature control. Dilute to the required concentration with sterile PBS buffer (pH 7.2, containing 5% trehalose).

RETRACTED

The first-level total score of the survey patient is as follows [8]:

(1) $$\begin{array}{c} E=\sum_{j=1}^{n}\frac{PQ}{i}. \end{array}$$

The total score of the second-level survey of patients is as follows [9]:

(2) $$\begin{array}{c} E=\sum_{j=1}^{n}\frac{PQ}{i}. \end{array}$$

*Lycium barbarum* polysaccharide extracted from the traditional Chinese medicine *Lycium barbarum* has a variety of biological effects, such as enhancing the body's immune function, antitumor, and antioxidation, and can also reduce bone marrow suppression in radiotherapy and chemotherapy. The statistics on medical treatment are [10]

(3) $$\begin{array}{c} \text{CONT}=\sum P\left(\text{EP}-0.5\right),\\ \text{CONT}=\sum P-{\text{CONT}}_{1,t}. \end{array}$$

The combination of traditional Chinese medicine polysaccharide with chemotherapy in the treatment of tumor patients showed that polysaccharide can not only produce obvious synergistic effect and enhance the immune function of tumor bearing body but also promote the development and differentiation of hematopoietic cells. For example, angelica polysaccharide can inhibit the proliferation of various malignant tumor cells in the blood system and promote the proliferation and differentiation of hematopoietic stem cells and progenitor cells. LBP can increase the number of nucleated cells and the number of granule/macrophage colonies in bone marrow and has the effect of endogenous CSF (colony stimulating factor).

The industrial characteristics of the Internet of Things are mainly reflected in the application field, and the intelligent application of the Internet of Things is realized through the combination of the application layer and industry requirements. In the medical field, the application of Internet of Things technology can realize smart medical care. In other words, the Internet of Things uses information recognition technologies such as sensors to build networks to realize smart medical services. The intelligent diagnosis of the Internet of Things is shown in Figure 1.

### 2.3. Experimental Method

#### 2.3.1. MTT Detection Method

Chemotherapy is one of the main means of malignant tumor treatment, but chemotherapy has a severe immunosuppression and side effects of hematopoietic inhibition; combining therapy with Chinese medicine polysaccharide can improve the body's immune function as a whole; on the basis of killing tumor cells, at the same time, chemotherapy can reduce side effects, and the role in the field of polysaccharide in tumor immunotherapy has grabbed wide attention and been favored.

RETRACTED

MTT colorimetric analysis is the relative quantification of the total number of liver fibrotic cells based on the optical density OD value determined by the enzyme plate. Normal pancreatic enzymes are used to digest cells that are growing well. In an appropriate amount of culture medium, the cells are blown to regenerate all cells. Next, according to the counting unit, the fibrotic cells inoculated on the 96-counting plate are combined with LBP-2 and LBP-3LB, respectively. The final concentrations of P-4 and LBP-5 were 400 and 800 *μ*g/mL, and 1200 and 1600 *μ*g/mL were set as well as the normal control group and the positive control group. The cells were incubated in the incubator for 24, 48, and 72 hours. The cells were collected in test tubes and washed twice with PBS, and finally PBS 2004 was added to each test tube. Use a flow cytometer to obtain 1 min under medium-speed conditions, and record the cell number, FSC, and SSC. The foundation of the Internet of Things center is now also the Internet. The network is expanded based on the Internet, and users exchange the expanded information. In other words, the Internet of Things is a new technology that connects sensors to the existing Internet. Today, smart medicine is an important development aspect in the medical field. The regional medical information platform is a regional medical service model established based on the information technology platform. It uses the Internet of Things technology to realize the interaction between patients and medical personnel, medical institutions, and medical equipment and provide health services. The medical IoT platform is shown in Figure 2.

#### 2.3.2. Effect of *Lycium Barbarum* Polysaccharides on Fibrosis

Establishment and combination of experimental model are as follows: when the state of cell proliferation is 80% to 90% fusion, the liver fibroblasts used in the selection experiment are all in a good state of reproduction. The 6 holes were inoculated with cells at a density of 2 × 10^4^/ml, and the glass cover for the immunofluorescence test was preinstalled with autoclaved glass. For different concentrations of LBP, different concentrations of LBP treat the cells for 24 hours. The effects of LBP culture with different concentrations on the proliferation of liver cancer cells were divided into 3 groups (5 *μ*mol/L, 10 *μ*mol/L, and 15 *μ*mol/L), and the concentration as a control group was 0 *μ*mol/L. Next, observe the inhibitory effects of different concentrations of LBP on the proliferation of hepatocellular carcinoma cells.

RETRACTED

#### 2.3.3. Effect of *Lycium Barbarum* Polysaccharide Combined with Positive Drug Fluorouracil on Killing Tumor Cells

According to the results of preliminary experiments, the concentration gradient of LBP is 200 mg/L and 400 mg/L, respectively. On the other hand, a solution of a fixed concentration of 1 *μ*mol/L was combined as a fluorouracil (5FU) group, and a control group and a mixed group of LBP and fluorouracil were set. Each group has 3 composite holes. After 48 hours, the cell morphology and changes of each drug group were observed through a microscope and photographed, and the relative inhibition rate of each drug concentration group on the cells was detected by the MTT method.

### 2.4. LBPs Affect the Viability of Liver Cells

The processing time of LBPs was set to 24 h. Take L-02 cells in logarithmic growth phase and incubate at 37°C for 24 h. The experiment sets up different concentrations and different molecular weight ranges, and each group has 6 multiple holes. Change the original medium, change into the medium containing different concentrations of LBPs (12.5, 25, 50, 100, and 200 *μ*g/mL), and culture for 24 h. The original medium was replaced, the control group was replaced with fresh medium, and the ethanol injury group was replaced with a medium containing 5% ethanol and cultured for 4 hours. Take the cultured cell supernatant for testing. Calculate cell viability according to the following formula [6]:

(4) $$\begin{array}{c} H=\frac{A_{G}-A_{K}}{A_{D}-A_{K}}\times 100\%. \end{array}$$

Calculate the consistency index [11] as follows:

(5) $$\begin{array}{c} \text{CI}=\frac{\lambda -N}{N-1}. \end{array}$$

There are *n* DMUs (decision-making units), *X* represents input indicators, *Y* represents output indicators, each DMU has m types of inputs and *s* types of output, and the weight coefficients *p* and *q* are used as variables to optimize the model for [12]

(6) $$\begin{array}{c} \max=\frac{\sum_{k=1}^{s}qkykvo}{\sum_{l=1}^{m}pixivo}=p\;d,\\ \text{s.t. }\frac{\sum_{k=1}^{s}qkykvo}{\sum_{l=1}^{m}jixiv\leq 1}. \end{array}$$

However, the antitumor mechanism of *Lycium barbarum* polysaccharides is not yet fully understood. Traditional Chinese medicine polysaccharide is a mixture of different molecular weight components extracted from traditional Chinese medicine. Current research shows that different molecular weight *Lycium barbarum* polysaccharide components may have different biological activities. Convert the above nonlinear fractional programming into the dual form of the equivalent linear programming [13]:

(7) $$\begin{array}{c} \text{s.t. }\sum_{v=1}^{n}\beta vxv+s^{-}=\beta x_{0},\\ \beta_{i}y_{i}+s^{+}=y_{o}. \end{array}$$

RETRACTED

### 2.5. In Vivo Experiment

In recent years, the ethanol gavage method has been widely used in animal modeling. Depending on the ethanol concentration, dosage, time in the stomach, and additives, modeling is very unstable, or animal mortality is high. In vivo antitumor studies on the direct cytotoxic effects of LBP on liver cancer cells and tumor suppression experiments in animals have confirmed that polysaccharides can hinder the growth of liver fibrotic cancer in mice.

LBPs medium is as follows: weigh 10 mg of LBPs sample powder correctly, add 20 mL of complete medium, prepare 0.5 mg/mL LBPs stock solution, and completely dissolve it at 40°C for 5 minutes. Then, the culture solution is uniformly mixed and sterilized using a sterilized microsphere membrane. Stored at 4°C, it is effective within 2 weeks. The mother liquor is completely diluted to the required concentration of the culture medium.

#### 2.5.1. In Vivo Activated Metabolism of Ascites Cells in Mice and Subcutaneous Fibrotic Cell Tumor Modeling

After microscopic observation of cells in a serum-free medium, 0.5 mL of cell suspension was prepared, all cell pellets were formed without exception, and male healthy mice of 229 g or more were used. In order to verify the activity, a cell suspension was prepared by injecting into the abdominal cavity of mice, and the size and mental state of the mice's abdomen were observed. For the third-generation mouse ascites, the third-generation mouse ascites has a good color and extracted 1 ml, respectively, extracted twice, mixed in the medium to dilute, and centrifuged to remove impurities; then add fresh serum-free medium to it, and count under a microscope. Constitutive cell concentration is 1 × 10^7^/mL; select 50 mice, sterilize the mouse right axillary area with 75% ethanol cotton swab, and inoculate 0.2 mL tumor cells (1 × 10^6^ cells); the tumor formation rate is 100%.

#### 2.5.2. Grouping of Experimental Animals and Methods of Administration

The successfully prepared subcutaneous fibroma model mice were randomly divided into 5 groups, and the classification and label were written in the rearing cage. They were cyclophosphamide group, LBP low-dose group, fibroma model group, joint CXCLIOLBP high-dose group, and *Lycium barbarum* polysaccharide. In the high-dose group, there are 10 animals in each group, but as a normal control group, there are 10 animals. Feed the animals on the third day after aseptic culture. In contrast, mice with liver fibrosis were given pelleted rat food and water before the 8th week. Add 2 mg/kg of *Lycium barbarum* (>95% purity; INDOFINE Chemical Company, Hillsborough, NJ) until the 8th week, and inject the *Lycium barbarum* solution with PBS and 5% Tween-80 (Solarbio, Beijing, China) compared. Observe for 14 days and continue medication. On the 15th day (at this time, some rats in the model group experienced cramps, fatigue, lack of food, etc.), the rats were anesthetized, blood was collected from the eyeballs, and the quality of the fibroids was determined by an analytical balance [14, 15]:

(8) $$\begin{array}{c} \text{BE}\left(1-\gamma \right)={\text{CI}}_{1,\gamma }+{\text{CI}}_{2,\gamma },\\ \text{BE}\left(1-\gamma \right)={\text{CI}}_{3,\gamma }+{\text{CI}}_{4,\gamma }+{\text{CI}}_{5,\gamma }. \end{array}$$

Here, *γ* represents the self-pay ratio [16].

RETRACTED

In essence, Euclidean distance represents the true distance between two points in a multidimensional space [17]:

(9) $$\begin{array}{c} d\left(x,y\right)=\sqrt{\left(\varphi \sum {\left(x_{{}_{i}}-y_{i}\right)}^{2}\right)}. \end{array}$$

The similarity expressed by Euclidean distance is [18]

(10) $$\begin{array}{c} \text{sim}\left(x,y\right)=\frac{1}{1+d\left(x,y\right)}=\frac{1}{1+\sqrt{\sum {\left(x-y\right)}^{2}}}. \end{array}$$

Pearson correlation coefficient is as follows [19]:

(11) $$\begin{array}{c} \varepsilon \left(x,y\right)=\frac{\mathrm{cov}\left(x,y\right)}{\sigma_{v}}. \end{array}$$

The cosine similarity represents the cosine value of the angle formed by the vector value of two triples in the vector space [20]:

(12) $$\begin{array}{c} \cos\left(\beta \right)=\frac{\sum x\sum y}{1+\sqrt{\sum x\sum y}}. \end{array}$$

Calculate the product *M* of each row element of the judgment matrix [21, 22]:

(13) $$\begin{array}{c} M=\prod_{J=1}a_{i,j}. \end{array}$$

Calculate the *n*th root of *M* [23]:

(14) $$\begin{array}{c} \bar{W}=\sqrt{M},\\ \bar{W}=\frac{\sqrt{M}}{\sum_{J=1}W}. \end{array}$$

LBP is a well-known traditional Chinese medicine or a tonic. It has a great protective effect on the liver and eyes. Calculate the largest characteristic root of the judgment matrix [24]:

(15) $$\begin{array}{c} \lambda =\sum_{i=1}\frac{{\left(AW\right)}_{i}}{nW_{i}}, \end{array}$$

(*AW*)_*i*_ represents the *i*th element of the vector AW [25].

#### 2.5.3. Observation of Staining

The wild balb/*c* mice (23–28 g) were divided into 2 groups (*n* = 4). Both the control group and the ZD group were fed normal food and water for 90 days. During this period, the wolfberry polysaccharide group was given 2 mg/kg of wolfberry red pigment every day for 90 days. Then, the serum ALT, AST, and TNF-*α* content were determined by the above-mentioned method, and the content of urea nitrogen (BUN) was determined using ADVIA2400 clinical instrument (Siemens Healthcare, Erlangen, Germany). The liver, heart, spleen, and kidney tissues of mice were stained with H&E to observe the damage.

RETRACTED

## 3. Results

LBP is the most important part of Lycium barbarum. Modern medical research results show that LBP has a wide range of biological effects, including resistance to aging, nerve protection, glucose metabolism control, blood lipid reduction, oxidation prevention, enhance immune regulation, and other effects.

The rats in the normal control group were 425 ± 28 grams by the end of the tenth week, and there was no death. Rats in the alcohol group were 286 ± 38 g at the end of the tenth week, which was significantly different from the normal control group. The masses of the 5% LBP group, 10% LBP group, and 10% CSH treatment group were 366 ± 34 g, 363 ± 37 g, and 371 ± 33 g at the end of the 10th week, respectively. There were 1 death, 3 deaths, and 1 death in each of the three treatment groups. At the end of the 10th week, the weight of the abstinence group was 326 ± 31 g, 9 died, and the mortality rate was as high as 32.14%. The conditions of the rats that died and died abnormally in the experiment are shown in Figure 3.

NAFLD is one of the leading causes of chronic liver injury worldwide. It is also strongly associated with other pathological conditions, including obesity, diabetes, cardiovascular disease, and metabolic syndrome symptoms. Although the pathogenesis of NAFLD has not been fully characterized, it is generally believed to be caused by IR, lipid metabolism dysfunction, OS, inflammation, and necrotic cell apoptosis. Each potential therapeutic strategy should target these pathological conditions in the liver. In the past few decades, nonpharmacological treatments for NAFLD have received increasing attention. These substances are widely available and have fewer side effects than drugs, and their therapeutic mechanisms and benefits have been demonstrated in many studies.

For each concentration of LBP, three repeated inhibition tests were done. In one well (the number of cells in each well is 125 × 10^3^), when the concentration of *Lycium barbarum* polysaccharide is 0 *μ*mol/L, the average number of uninhibited cells is 124.00 × 10^3^. The effect of fibrotic cell inhibitory concentration is shown in Table 1.

LBP is a famous Chinese medicine or tonic, which has shown great protective effect on liver and eyes. Mild to moderate abnormalities of ALT and/or AST are sometimes the only abnormal manifestations of NAFLD. Therefore, ALT and AST can be regarded as indicators of abnormal liver function. In this study, LBP was dry ALT and AST in pregroup were lower than those in NAFLD group, suggesting that LBP has protective effect on liver cells.

RETRACTED

The immune system plays an important role in fighting tumors and fighting infections. Therefore, it is important to reduce the side effects and immunosuppression of chemotherapy drugs in the bone marrow and to protect the body's immune function. At present, biologics represented by stimulating factor (G-CSF) have various degrees of side effects in clinical use and even cause secondary tumors. People are strongly demanding to find new reagents for chemotherapy. The effect of suppressing the number of fibrotic cells is shown in Table 2.

Compared with the normal control group, the levels of lipofuscin and LPO in drosophila salivary gland cells in the group supplemented with LBP extract significantly decreased, suggesting that LBP can inhibit the production of ROS, reduce the effect of LPO, and protect cells to a certain extent. Clinical trials have also found that LBP can also increase serum antioxidant levels while reducing the formation of lipid peroxides.

*Lycium barbarum* polysaccharides can significantly inhibit the proliferation activity of HCCLM3 in in vitro experiments. At different LBP concentrations (0 *μ*mol/L, 5 *μ*mol/L, 10 *μ*mol/L, and 15 *μ*mol/L), the inhibition rates are 0.80%, 20.06%, 35.44%, and 55.39%, respectively. LBP concentration of 5 *μ*g/mL, 1 *μ*g/mL, and 2 *μ*g/mL (1.008 ± 0.090 *μ*g/mL versus 1.473 ± 0.083 *μ*g/mL, 1.063 ± 0.050 *μ*g/mL versus 1.473 ± 0.083 *μ*g/mL, and 1.040 ± 0.078 *μ*g/mL versus 1.473 ± 0.083 *μ*g/mL, *P* < 0.05) had a greater impact on cell viability. The inhibition rate at different LBP concentrations is shown in Figure 4.

Radiotherapy is also the traditional method of liver cancer treatment. With the improvement of radiotherapy technology, radiotherapy plays an active role in palliative treatment of liver cancer. In recent years, molecular targeted therapy and immunotherapy have also been gradually applied in the treatment of liver cancer.

The western blot experiment is the average of three experimental results. The three experimental conditions are exactly the same. The VEGF protein concentration of the control group is set to 1 *μ*mol/L. In the results of this experiment, the ratio of the concentration of VEGF protein is 0.71, 0.57, and 0.27. In the second experiment, the ratio of VEGF protein concentration was 0.88, 0.59, and 0.47. Surgery is mainly the preferred treatment method for liver fibrosis including liver resection and transplantation. Surgical resection of the liver can effectively improve the survival rate of 50% of tumor patients, but surgical treatment is mainly suitable for early-stage patients. There are requirements for the size and nature of the tumor, as well as the status of patients with obvious heart and lungless patients, and no renal dysfunction is required. The results of the western blot experiment are shown in Figure 5.

RETRACTED

However, the effect of any current treatment or drug therapy is not satisfactory, which is also the main reason for the high death rate of liver cancer. At present, comprehensive treatment is a new strategy for the treatment of liver cancer in different stages of development, such as chemotherapy after surgical resection or liver transplantation to prevent recurrence. Or a combination of radiation and chemotherapy often works better than treatment alone.

When the LBP concentration is set to 0 *μ*mol/L, the protein concentration of VEGF is 1. When the LBP concentration is 5 *μ*mol/L, 10 *μ*mol/L, and 15 *μ*mol/L, the protein concentration of VEGF is 0.75 ± 0.05, 0.56 ± 0.03, and 0.36 ± 0.06 *μ*mol/L, respectively. The protein concentration of VEGF is shown in Figure 6.

However, polysaccharide from traditional Chinese medicine is a mixture composed of a series of polysaccharide components with different molecular weight, which may have different biological activities. The main active components and mechanism of antitumor and immunomodulatory effects of LBP have not been clear, which also needs further study.

At present, the research on the modern molecular level of traditional Chinese medicine to prevent and treat ALD is still not deep enough, and the lack of exploration in signal transduction pathways, genome, and proteomics makes it difficult for traditional Chinese medicine to become the universal medical language in the world. The activity levels of ALT and AST in the cell culture medium of the ethanol injury group were 3.10 and 3.25 times that of the control group, respectively, and the difference was statistically significant (*P* < 0.01). The results of this experiment show that the ethanol-induced hepatocyte injury model was successfully constructed. The cell culture condition of ethanol damage is shown in Figure 7.

*Lycium barbarum* polysaccharide (LBP) extracted from Chinese medicine *Lycium barbarum* has many biological effects, such as enhancing immune function, antitumor, and antioxidation and alleviating bone marrow inhibition by radiotherapy and chemotherapy. Existing studies suggest that LBP has the functions of antitumor and protective agent of chemotherapy and has the potential to reduce the immune toxicity of adriamycin and enhance its anti-liver cancer effect.

Compared with the control group, the cell viability of the ethanol injury group was significantly reduced (*P* < 0.01), and the cell viability was 66.48% ± 4.30%. The cell viability of the ethanol injury group is shown in Figure 8.

RETRACTED

After 24 hours of plating, the cells of each group showed adherent growth, and the cell status was good. 48 hours after the addition of the drug, the low-dose wolfberry polysaccharide 200 mg/mL combination control group did not change significantly compared with the cell morphology under the microscope, while some cells in the 400 mg/mL group rounding, the shrinking, and rounding of 800 mg/mL group showed that the number of apoptotic cells increased. At high doses of *Lycium barbarum* polysaccharide, most of the adherent cells showed reduced volume and rounded growth, and the number of cells was very small. The cell growth is shown in Figure 9.

The results of MTT showed that each group of drugs had a certain inhibitory effect on cells and was dose-dependent. The inhibition rates of the *Lycium barbarum* polysaccharide group alone (200 mg/L, 400 mg/L, 800 mg/L, and 1000 mg/L) were 9.23%, 22.80%, 36.84%, and 76.25%, respectively. The MTT results are shown in Table 3.

Relative to the tumor quality of the model group, the low-dose LBP, high-dose LBP, LBP + CXCLIO, and CTX medication groups all showed a certain tumor inhibition trend, and the inhibition rates were 37.83%, 12.50%, 16.11%, and 59.20%, respectively. The changes of tumor mass in different groups are shown in Table 4.

The results of flow cytometry showed that the Th1/Th2 ratio of the LBP combined with CXC110 group increased significantly to 6.12 ± 3.89, while the model group was only 0.87 ± 0.42. The change of Th1/Th2 ratio is shown in Table 5. The effects of different molecular weight LBP components on the growth of mouse liver cancer xenografts in vitro experimental results show that different molecular weight LBP components have different effects on the proliferation of mouse H22 liver cancer cells and the function of lymphocytes and macrophages. However, the physiological environment in vivo is more complicated than the experimental environment in vitro. The inhibition of polysaccharides in vitro on fibrotic cells and the regulation of immune cell function cannot fully reflect its antitumor and immunoregulatory effects in vivo.

Among them, amino acid aminotransferase (ALT), aspartate aminotransferase (AST), lactate dehydrogenase (LDH), ALT, and AST can be regarded as indicators that reflect abnormal liver function. In this experiment, ALT and AST in the LBP intervention group were lower than those in the NAFLD group, suggesting that LBP has a protective effect on liver cells. Compared with the ethanol injury group, the ALT, AST, and LDH activities of the 25 and 100 *μ*g/mL LBPs groups were significantly reduced (*P* < 0.05). The results showed that LBPs can inhibit the release of ALT, AST, and LDH in hepatocytes induced by ethanol. Make full use of postgenomics ideas and modern molecular biology technologies such as biochips, establish the concept of transformation mode related to genomics and proteomics and traditional Chinese medicine, link the modernization of traditional Chinese medicine research with life sciences, and make it a clear mechanism of action; the material basis is clear, and it is a modern and vigorous drug that is universally accepted internationally. The activities of ALT, AST, and LDH are shown in Figure 10.

RETRACTED

## 4. Discussion

Liver fibrosis (LF) is a general pathological feature of most chronic liver diseases and is an inevitable stage of the onset of liver cirrhosis. Because LF can be reversed, research on the treatment of liver fibrosis has become a hot topic. Because it is difficult to overcome the toxicity and side effects of western medicine treatment, it is difficult to be widely used in clinics. TCM has a long history in the treatment of liver fibrosis. In recent years, people have conducted extensive and detailed studies on the effective ingredients of many TCM extracts for liver fibrosis [26].

External pollutants (heavy metals such as cadmium, chromium, arsenic, organic poisons such as carbon tetrachloride, etc.) may cause chemical liver injury (CLI). CLI appears as fatty liver, hepatitis, fibrosis, and even liver cancer and has attracted the attention of researchers in the fields of toxicology, nutrition, and food science. Mitochondria have their own genome, but their synthesis and function require nuclear-encoded proteins. Under the action of various transcription factors and core collagen, these proteins regulate the transcription of nuclear and mitochondrial genetic factors, and regulate body temperature, energy intake, and exercise capacity. LBP of different molecular weights will reduce cell viability and may hinder the proliferation of fibrotic cells. LBP-3 has the most important effect. Further studies have shown that LBP-3 has a dependent effect on the dosage of S phase arrested liver fibrotic cell cycle, reduces the mitochondrial membrane potential, and may cause liver fibrotic cell death [27].

Liver cancer is formed under the combined action of various factors. *Cancer* cells proliferate and metastasize through various methods or signal transmission pathways. Due to the complexity of the microenvironment of tumor tissues, a single treatment method cannot effectively control the onset of liver cancer. Therefore, exploring multiple methods and multiple drugs combined therapy has become a new strategy for the treatment of liver cancer. For mild alcoholic fatty liver and alcoholic hepatitis, control of alcohol and active treatment can restore the original state, but if not treated in time, all types of ALD will eventually lead to alcoholic liver cirrhosis, gastrointestinal bleeding, and development due to shock of all kinds of infections and other complications of liver cirrhosis. This is also the main cause of death in ALD patients [28].

RETRACTED

Extrinsic chemicals are mainly produced by liver metabolism, and liver toxicity is mainly related to the formation of active metabolites. Normally, the liver is detoxified through phase I and phase II. When the cellular defense mechanism is disrupted, exogenous chemicals are usually metabolized by phase I phosphate P450 enzyme involved in oxidation, reduction, or hydrolysis, producing a large number of electron affinity groups and free radicals. In addition, the covalent protein binding produced by active metabolites may also cause immune damage.

LDH is widely present in the cytoplasm of hepatocytes and can indirectly evaluate the survival rate of cells and the degree of damage to cell membranes. Reducing the emission of transaminase and LDH is an important indicator for testing the preventive and therapeutic effects of natural ingredients on liver dysfunction. The intervention of polysaccharides can reduce the release of ALT, AST, and LDH in liver cells. Therefore, by measuring the release of liver kinase and LDH in cell culture fluid, it can reflect the degree of damage to liver cells caused by ethanol and antifibrotic drugs [29].

In recent years, with the deepening of experimental research on the prevention and treatment of medical liver fibrosis and the research process mechanism, from the perspective of the effective ingredients of Chinese medicine, the preparation of single drugs and compounds has a good prospect, but from the perspective of pathology in the classic enzyme studies, most of the biochemistry, histochemistry, immunohistochemistry, radioimmunology, and so on show the mechanism of drugs by observing the pathological changes of the liver, the enzyme spectrum, and the cells of the liver [2].

## 5. Conclusion

This study found that LBPs can inhibit liver cell oxidative stress damage, and the Nrf2 pathway is a key transcription factor involved in liver cell metabolism and detoxification. Several downstream antioxidant enzymes are important components of the liver's antioxidant system. Excitogen plays a key role in maintaining cell oxidation homeostasis. Therefore, in order to explore the protective mechanism of LBPs on chemical hepatocyte damage caused by oxidative stress, this study used western blot to detect the effect of LBPs intervention on the expression of related proteins in the Nrf2 pathway of hepatocytes. The antitumor effect of *Lycium barbarum* polysaccharide has been confirmed. Research in recent years has shown that the biological activity of polysaccharide may be related to its chemical structure and molecular weight. In vitro experiments in this study have also confirmed that LBP has four different molecular weight soluble *Lycium barbarum* polysaccharide components. Strongly inhibit the proliferation of mouse liver cancer cells and enhance the function of immune cells. In this study, through in vivo tumor suppression experiments, it was found that LBP can significantly inhibit the growth of liver cancer transplanted tumors in mice, and its antifibrotic tumor effect is significantly stronger than other molecular weight polysaccharide components. The effect of *Lycium barbarum* polysaccharide on transaminase does not show a linear dose-effect relationship with its dosage. The exact mechanism is not fully understood. With the development of medical immunology and molecular biology technology, the antitumor immune mechanism of polysaccharides will be more in depth. Liver fibrosis is a challenge in the new era, and it is the key to preventing and treating patients progressing to end-stage liver disease. Liver fibrosis and end-stage liver disease are problems affecting the world. Liver fibrosis determines the morbidity and death of patients with liver disease and causes liver failure and is related to the occurrence of primary liver cancer. In the process of liver fibrosis caused by various reasons, immune factors have played an important role. Various damage stimuli act on the liver, leading to the activation or inhibition of immune cells and the production of a variety of cytokines. The disorder of these cells and their cytokines promotes or inhibits the formation and development of liver fibrosis. However, these immune factors have not been fully elucidated, and further elucidation of these problems will provide us with various methods and basis for blocking the formation and development of liver fibrosis, which will help to treat this kind of diseases in a reasonable and effective clinical way. In the future, more drugs for treating liver fibrosis need to be studied.

RETRACTED

## Figures and Tables

**Figure 1:** Intelligent diagnosis of the Internet of Things.

**Figure 2:** Medical Internet of Things platform.

**Figure 3:** Conditions of rats executed and those that wrongfully died in the experiment.

**Figure 4:** Inhibition rate at different LBP concentrations.

**Figure 5:** Results of the western blot experiment.

**Figure 6:** Protein concentration of VEGF.

**Figure 7:** Situation of ethanol-damaged cell culture.

**Figure 8:** Cell viability in the ethanol damage group.

**Figure 9:** Cell growth.

**Figure 10:** ALT, AST, and LDH vitality.

**Table 1:** Effect of the fibrotic cell inhibitory concentration.

LBP concentration (*μ*mol/L)	First time	Second time	Third time	Average value
0	124.2	124.4	123.4	124.00
5	101.9	99.9	98.0	99.93
10	83.4	77.6	81.1	80.70
15	56.0	59.0	523	55.76

**Table 2:** Effect of fibrotic cell number inhibition.

LBP concentration (*μ*mol/L)	Number of uninhibited cells	Number of suppressed cells	Total	Inhibition rate (%)
0	124.00	1.00	125.00	0.80
5	99.93	25.07	125.00	20.06
10	80.70	44.30	125.00	35.44
15	55.76	69.24	125.00	55.39

**Table 3:** MTT bear fruit.

Group	LBP (mg/L)	5FU (umo1/L)	Inhibition rate (%)
Blank control group	0	0	0
LBP1 group	200	0	9.23 ± 0.20
LBP2 group	400	0	22.80 ± 5.83
LBP3 group	800	0	36.84 ± 2.30
LBP4 group	1000	1	76.25 ± 8.23
5FU group	0	1	34.15 ± 0.73
Combine 1 group	200	1	45.15 ± 1.13
Combine 2 groups	400	1	81.10 ± 1.53

**Table 4:** Tumor mass in the different groups.

Group	N	Average tumor mass (g)	Tumor inhibition rate (%)
Normal	10	—	—
Model	7	3.04 ± 1.06	—
CTX	9	1.24 ± 0.84	59.20
Low-dose LBP	10	1.89 ± 1.21	37.83
High-dose LBP	8	2.66 ± 1.68	12.50

**Table 5:** Th1/Th2 ratio change.

Group	Th1 (%)	Th2 (%)	Th1/Th2
Normal	10.61 ± 4.72	7.75 ± 3.52	1.52 ± 0.59
Model	12.35 ± 7.74	21.48 ± 23.23	0.87 ± 0.42
CTX	4.05 ± 3.16	2.83 ± 2.05	2.01 ± 1.99
Low-dose LBP	28.38 ± 21.98	7.71 ± 5.24	6.05 ± 7.83
High-dose LBP	18.58 ± 7.61	18.88 ± 13.69	2.48 ± 2.93

## Data Availability

The data that support the findings of this study are available from the corresponding author upon reasonable request.
